# Solanum Procumbens-Derived Zinc Oxide Nanoparticles Suppress Lung Cancer In Vitro through Elevation of ROS

**DOI:** 10.1155/2022/2724302

**Published:** 2022-09-13

**Authors:** Ibrahim Ibrahim Abdel Aziz, Almaimani A. Riyad, Almasmoum A. Hussian, Ghaith M. Mazen, Moorthy Kannaiyan

**Affiliations:** ^1^Department of Pharmacology and Toxicology, Faculty of Medicine, Umm Al-Qura University, Makkah, Saudi Arabia; ^2^Department of Biochemistry, Faculty of Medicine, Umm Al-Qura University, Makkah, Saudi Arabia; ^3^Department of Laboratory Medicine, Faculty of Applied Medical Sciences, Umm Al-Qura University, Makkah, Saudi Arabia; ^4^Department of Medical Laboratory Science, School of Pharmacy and Medical Laboratory Science, Institute of Health, Bule Hora University, Bule Hora, Ethiopia

## Abstract

Lung cancer is one of the cancers with high mortality rate. The current therapeutic regimens have only limited success rate. The current work highlights the potential of *Solanum procumbens*-derived zinc oxide nanoparticle (SP-ZnONP)-induced apoptosis in A549 lung cancer cells. Synthesized nanoparticles were confirmed by UV-Vis spectrophotometry, X-ray diffraction (XRD), dynamic light scattering analysis (DLS), scanning electron microscopy (SEM), Fourier transform infrared (FT-IR), and photoluminescence analysis. Lactate dehydrogenase (LDH), cytotoxicity, and cell viability assays revealed that the SP-ZnONP caused the cell death and the inhibition concentration (IC_50_) was calculated to be 61.28 *μ*g/mL. Treatment with SP-ZnONPs caused morphological alterations in cells, such as rounding, which may have been caused by the substance's impact on integrins. Acridine orange/ethidium bromide dual staining revealed that the cells undergo apoptosis in a dose-dependent manner, which indicates the cell death. Furthermore, reactive oxygen species (ROS) were examined and it was shown that the nanoparticles elevated ROS levels, which led to lipid peroxidation. In short, the SP-ZnONPs increase the level of ROS, which in turn causes lipid peroxidation results in apoptosis. On the other hand, the SP-ZnONPs decrease nitric oxide level in A549 cells in a dose-dependent manner, which also supports the apoptosis. In conclusion, SP-ZnONPs would become a promising treatment option for lung cancer.

## 1. Introduction

Lung cancer is one of the leading causes of cancer-mediated deaths worldwide [1]. Although a variety of treatment strategies such as surgery, radiation therapy, chemotherapy, and targeted therapy has been followed to treat lung cancer, the outcome is poor [2]. Targeted therapy using inhibitors of angiogenesis, KRAS, EGFR, AKL, and BRAF has also been widely used to treat lung cancers. In spite of a variety of targeted therapeutic agents, the success is very much limited. Therefore, we explored the possibility of *Solanum procumbens*-derived zinc oxide nanoparticle (SP-ZnONP) for treating lung cancer.

Experimentally, zinc oxide nanoparticles (ZnONPs) have already been shown to be effective in alleviating the cancer. Particularly, ZnONPs have become a one of the treatment options for cancer due to several reasons such as biocompatibility, selectivity, ease of synthesis, ability to induce cytotoxicity, and high surface area to volume ratio [3]. In addition, ZnONPs efficiently involve in the redox reaction system led to elevate the reactive oxygen species (ROS) [4]. Most importantly, selective cytotoxicity is enhanced by ZnONPs since ROS and related signalling molecules are produced more in cancer cells due to rapid metabolic rate compared with normal cells [5]. Recent reports suggest that ZnONPs are also effective in reducing the stemness of cancer stem cells in breast cancer [6].

Solanum procumbens Lour. (Solanaceae) is a tropical plant found in South East China, Vietnam, Thailand, Laos, and Hainan. It has been widely used in traditional and folk medicines. Formulations containing this plant extract have been used for the treatment of ailments such as rheumatism, pain, detoxification, hepatitis, and cirrhosis. [7]. Spirosolane alkaloids, pregnane steroids, and steroidal saponins are major constituents of Solanum procumbens extracts [8]. In the present work, we prepared Solanum procumbens extract and used for the preparation ZnONPs and evaluated its potency to treat lung cancer.

## 2. Materials and Methods

### 2.1. Plant Extract Preparation

The fresh leaves of *Solanum procumbens* (SP) were collected and thoroughly washed with distilled water to eliminate dirt particles and prevent contamination. With the help of mortar and pestle, around 5 g of *Solanum procumbens* leaves was prepared into fine paste and blended in 500 mL of distilled water and then heated at 70°C for 30 minutes. Further filtration of extract was carried out by muslin cloth followed by Whatman filter paper. The filtered plant extract stored at 5°C for further applications.

### 2.2. Synthesis and Characterization of Green-Synthesized ZnONPs [9]

An aqueous solution of 95 ml zinc chloride (0.01 M) was mixed with 5 mL of plant extract of *Solanum procumbens.* The mixture was kept in a shaking incubator for 1 hour at 70°C with 150 rpm. At the end of the reaction, a white precipitate settled at the bottom of the flask. The supernatant was removed from the white precipitate and transferred to a 1.5-mL centrifuge tubes. The samples were washed with distilled water through centrifugation at 3000 rpm for 30 minutes and repeated process thrice to remove impurities completely and dried in a hot air oven at 90°C. The dried product was then ground into a powder using mortar and pestle and calcined at 500°C for 2 hrs. Finally, the resultant annealed powder stored in an airtight glass vial and labelled as SP-ZnONPs. The optical properties synthesized SP-ZnONPs were analysed using UV-Vis and photo-luminescence spectroscopy. Its physical nature and particle size were obtained by XRD and DLS. Furthermore, shape and surface morphology were identified using TESCAN VEGA3 scanning electron microscopy (SEM). Fourier transform infrared (FTIR) spectroscopy was used to confirm the existence of functional groups in the synthesized nanoparticles.

### 2.3. Cytotoxicity Assay

The mitochondrial function was investigated by MTT(3-(4,5-dimethylthiazol-2-yl)-2,5-diphenyltetrazolium bromide) assay as described by Mossman, 1983, with slight modification. [10] The 96-well plates were seeded with A549 cells (5 × 10^4^ cells/well) and incubated for 24 hours and treated with SP-ZnONPs at various concentrations (5–200 *μ*g/mL) for 48 hours. 15 *μ*L of MTT solution (5 mg/mL PBS) was added to cells and incubated at 37°C for 4 hours. After removing supernatant, thin soluble formazan product was dissolved in DMSO and shaken up for 10 min at room temperature and analysed by microplate reader at 490 nm and 630 nm. Untreated cells considered as negative control. Inhibition of cells was calculated by % Inhibition = {1- [*A*_490_—*A*_630_ (Treated)/*A*_490_—*A*_630_ (control)] × 100}.

### 2.4. Cell Viability by Trypan Blue Exclusion Assay

The lethality of SP-ZnONPs on A549 cells was assessed by the trypan blue exclusion test (Crowley et al. ) [11]. Cells were seeded in 6-well plates with different concentrations of SP-ZnONPs as 10, 20, 30, 40, 50, 60, 70, 80, 90, and 100 *μ*g/mL for 24 h of exposure in a humidified incubator (5% CO_2_, 37°C). Thereafter, cells were trypsinized and resuspended in equal volume of culture medium and trypan blue stain. Viable (unstained) and nonviable (blue-stained) cells were counted using a haemocytometer to calculate the total number of live and dead cells.

### 2.5. Morphometric Analysis

The morphological changes of apoptotic cells were analysed by the method reported elsewhere [12] with slight modifications. After seeding 5 × 10^5^ cells, it was incubated for 24 hours and treated with three concentrations of SP-ZnONPs (50, 60, and 70 *μ*g/mL) for another 24 hours. The medium was removed, and cells were washed with PBS and observed for morphological changes of the treated cells under inverted phase contrast microscope at 20X magnifications.

### 2.6. Analysis of Dual Staining

The apoptotic cell death analysis was carried out by fluorescence microscope combining the methods by Reference [13, 14]. SP-ZnONPs-treated A549 cells were investigated by AO/EB fluorescence staining techniques for morphological alterations due to apoptosis. 1 × 10^5^ cells were seeded in a 12-well plate over sterile coverslips coated with Poly-*L*-Ornithine solution and incubated in a CO_2_ incubator overnight at 37°C for 24 hours. After removal of medium, the cells were treated with different concentrations of SP-ZnONPs (50, 60, and 70 *μ*g/mL and control) and incubated for 48 hours. The medium was removed and washed with PBS. Coverslips were washed with 1 mL 1X DPBS and stained with 200 *μ*L staining solution (1 mL of ethidium bromide (50 *μ*g/mL) and 20 *μ*L of acridine orange (20 *μ*g/mL)) for 10 minutes. The staining solution was removed and observed under fluorescence spectroscopy with excitation at 560/40 nm and emission at 645/75 nm for EtBr and excitation 470/40 and emission 525/50 for acridine orange and recorded using ImageJ software.

### 2.7. ROS Estimation

The NBT reduction assay was performed to estimate the ROS, which is slightly modified version of Abdulhamid and Morgan method [15]. 1 × 10^5^ cells/mL cells were seeded and incubated for 24 hours. SP-ZnONPs were then added onto the appropriate well at different concentrations such as 50, 60, and 70 *μ*g/mL and incubated for 24 hours and washed with PBS twice. 100 *μ*L of 0.1% NBT solution was added and incubated for 1 hour followed by 70% of methanol thrice. About 120 *μ*L of 2 M potassium hydroxide (KOH) with 120 *μ*l of DMSO was added and read using plate reader at 630 nm, and the DMSO was considered as blank.

### 2.8. Determining Nitric Oxide Concentration

Nitric oxide concentration was estimated according to the method explained by Grdovicet al. [16]. 100 *μ*l of (100 *μ*M) of nitrite solution was added to each well of 96-well plate to perform nitrite standard reference curve. To achieve desired concentration, a series of dilutions was performed (100, 50, 25, 12.5, 6.25, 3.13, and 1.56 *μ*M). The equilibration of sulphanilamide and NED solutions was performed at room temperature (15–30 minutes). 50 *μ*L of each (various concentrations such as 50, 60, and 70 *μ*g/mL of SP-ZnONPs-treated solutions) was added to experimental supernatants to the wells as duplicates. Further 50 *μ*L of the 1% sulphanilamide dissolved in 5% phosphoric acid was added to samples in dilution series as a standard. The reaction mixture was incubated for 5–10 minutes at room temperature and protected from light followed by 50 *μ*L of the 0.1% NED solution to all wells. The absorbance was measured within 30 minutes after the colour generation at 520 nm and 550 nm.

### 2.9. Quantification of Lipid Peroxidation

The lipid peroxidation was quantified through spectrophotometrically by the complex formation of [17] malondialdehyde with thiobarbituric acid. The cells at the density of 1 × 10^4^ were seeded and incubated for 24 hours and treated with various concentrations of SP-ZnONPs (50, 60, and 70 *μ*g/mL). The treated cells were taken, and the pellet was washed and redispersed into 0.2 mL of 8.1% SDS. Then, 1.5 mL of 20% acetic acid was added to this suspension and incubated for 10 minutes, and then added with 1.5 mL of 0.8% TBA buffer and 0.7 mL of distilled water. This reaction mixture was incubated at 95°C for 1 hour, cooled to 25°C, and subjected to centrifugation at 5000 rpmg for 15 minutes to remove cell debris. Finally, the absorbance spectra were recorded at 532 nm along with blank and control.

### 2.10. Measurement of LDH Activity

LDH activity was determined according to the slightly modified version of reported method [18]. The cells at the density of 1 × 10^4^ cells/well were seeded and incubated for 24 hours followed by treatment with various concentrations (50, 60, and 70 *μ*g/mL) of SP-ZnONPs. The supernatant of treated cells was separated by centrifugation at 4°C for 10 minutes at 3000 rpm. LDH leakage was measured in a 3.0 mL of reaction mixture (28 mL of 100 mM potassium phosphate buffer pH 7.5, 1.20 mL of 100 mM sodium pyruvate, and 0.8 mL of 13.1 mM NADH; 3 mL of mixture incubated at 37°C for 3 minutes) with 10 *μ*L supernatant. The absorbance was recorded at 1-minute interval up to 4 minutes at 340 nm. The amount of LDH released is expressed as U/mg of protein in culture media.

### 2.11. Statistical Analysis

The triplicate results of all experiments were subjected to statistical analysis using GraphPad Prism version 5.1. Data are presented as mean ± standard deviation by one-way analysis of variance (ANOVA) with Tukey's multiple t-test.

## 3. Results

### 3.1. Characterization of Green-Synthesized SP-ZnONPs

#### 3.1.1. UV-Visible Spectroscopy

Zinc ions in the solution converted into *o* zinc oxide due to the presence of secondary metabolites in plant extract. Here, the plant extract acts as a pH altering and stabilizing agent. The UV-Vis absorption spectrum of SP-ZnONPs shows peak at 372 nm, which is around 7 nm red shifted compared with the bulk ZnO that shows peak at 365 nm, which confirms the formation of SP-ZnONPs (Figure 1).

#### 3.1.2. XRD and DLS Analysis

The generation of SP-ZnONPs was confirmed by XRD with Bragg's reflection, which corresponds to (100), (002), (101) (102), (110), (103), (200), (112), (201), (004), and (202) (Figure 2) with average particle size of 52 nm. Further DLS analysis revealed average particle size of 154 nm as shown in Figure 3. The reason for the higher particle size observed in DLS than that of in XRD is due to its hydrodynamic character.

#### 3.1.3. Photoluminescence Analysis

Figure 4 shows photoluminescence spectrum of SP-ZnONPs with the excitation wavelength at 325 nm.

### 3.2. SEM Analysis of Nanoparticles

The scanning electron microscope (SEM) was used to characterize the morphology of green-synthesized SP-ZnONPs.  Figure 5 shows the SEM image of the prepared nanoparticles, which reveals that the nanoparticles are well distributed and, more significantly, that they have an aggregative nature.

### 3.3. FTIR Analysis

FTIR spectrum of Solanum procumbens extract and SP-ZnONPs was shown in Figure 6(a) and 6(b), respectively. The peak at 495 cm^−1^ in the Figure 6(b) confirms the presence of SP-ZnONPs because the peak between 400 and 600 cm^−1^ region responsible for stretching frequency of Zn–O bond in ZnONPs. The broad peak at 3436 cm^−1^ in both Figures 6(a) and 6(b) confirms the presence of alcohol and phenolic OH groups; it is clearly understood that phenols and alcohols present in the extract are caped with the nanoparticles.

### 3.4. Cytotoxicity Assay

In order to understand the ability of green-synthesized SP-ZnONPs on the cancer treatment, these nanoparticles are treated with A549 lung cancer cell line. In the MTT assay, a dose-dependent cell death was observed. At a higher concentration of the nanoparticles (200 *μ*g/mL), 100% of cell death is observed. At lower concentrations (5 *μ*g/mL), there were little effects on cells in terms of viability (Figure 7). Overall, there was a dose-dependent cell death observed with green-synthesized nanoparticles and the IC_50_ was calculated to be 61.28 *μ*g/mL. With this result, it is apparent that the nanoparticle is highly effective in inhibiting the cell proliferation of lung cancer cells.

### 3.5. Cell Viability Assay

The relative proportion of viable cells was analysed using trypan blue exclusion assay. At 10 *μ*g/mL concentration, there were 93% cell viability, and at 100 *μ*g/mL, a majority of cells were died (Figure 8). 50% of cell death was observed at 60 *μ*g/mL concentration, which surprisingly correlates with value found in MTT assay.

### 3.6. Morphological Analysis

As the nanoparticles induced cell death in a dose-dependent manner, the cells were visualized under microscope to check for any morphological changes. Consistent with earlier observations, there was a dose-dependent reduction in cell number when observed under microscope. In addition, there is a significant difference in the morphology of A549 cells observed under the microscope. There is a significant decrease in the number of cells on treatment with SP-ZnONPs at concentrations of 50, 60, and 70 *μ*g/mL compared with untreated cells. The morphological changes observed in treated cells include cell shrinkage and cell rounding (Figure 9(b)–9(d)). The normal architecture was observed in untreated cells (Figure 9(a)). 5 *μ*g/mL of standard control cisplatin showed an increased number of apoptotic cells (Figure 9(e)).

### 3.7. Dual Staining-Acridine Orange/EtBr Staining

The signs of apoptosis were evaluated using acridine orange/ethidium bromide dual staining. Morphological changes in cancer cell nuclei were observed by fluorescent microscopy, which differentiates between normal and apoptotic cells. The observations in the fluorescent micrograph reveal that the death of A549 cells increased at high dosage of SP-ZnONPs (70 *μ*g/mL) (Figure 10(d)) compared with untreated cells (Figure 10(a)); it is showing that greater number of apoptotic cells were observed with blebbing of cell membrane and chromatin condensation in a dose-dependent manners. At 50 *μ*g/mL concentration, cells with various morphologies with varying stages of apoptosis such as healthy cells and early apoptotic cells could be observed. Necrotic cells could also be observed rarely (Figure 10(b)). In the 60 *μ*g/mL concentration, all types of cells such as viable cells, early apoptotic cells, and late apoptotic cells including some necrotic cells were evidenced (Figure 10(c)). Relative proportion of viable cells decreased with higher incidence of early and late apoptotic cells in 70 *μ*g/mL concentration (Figure 10(d)).

### 3.8. Estimation of ROS Level

The ROS level in A549 cell line was evaluated using NBT reduction assay. 50, 60, and 70 *μ*g/mL concentrations of SP-ZnONPs were chosen for assay and treated with the A549 cells. A dose-dependent significant increase in ROS level with increasing concentration of SP-ZnONPs was observed (*P* value > 0.0001). ROS level is apparently increasing when exposing SP-ZnONPs on A549 cells (Figure 11).

### 3.9. Nitric Oxide Assay

Cellular nitric oxide level decreased with increasing concentration of SP-ZnONPs. Upon exposing SP-ZnONPs at a concentration of 50, 60, and 70 *μ*g/mL on the A549 cell line, there is a dose-dependent decrease in nitric oxide (NO) level (Figure 12). When compared with control cell line, NO level in treated cells was significantly decreased. The decrease NO level was further studied through the complete cellular mechanism of NO generation. Results are expressed as mean and SD. Results were subjected to one-way ANOVA (Tukey multiple comparison test) and showed significant difference between control and treated cells. Treated cells showed high significance compared with control cells (*P* < 0.0001).

### 3.10. Determination of Lipid Peroxidation Activity

Thiobarbituric acid reactive substance (TBARS) assay was performed to quantify the extent of lipid peroxidation induced by the exposure of SP-ZnONPs on to the A549 cell line. The concentrations of 50, 60, and 70 *μ*g/mL of SP-ZnONPs were chosen for the quantification. There was a significant dose-dependent increase in the lipid peroxidation levels (Figure 13). This evaluation revealed that the nanoparticles were quite efficient in elevating the lipid peroxidation. Treated cells show higher significance compared with control cells (*P* < 0.0001).

### 3.11. Measurement of Lactate Dehydrogenase Activity

Lactate dehydrogenase activity (LDH) signifies the cell lysis. Upon cell lysis, the enzyme is exposed to the outside of the cell. Upon treating the A549 cancer cell lines with 50, 60, and 70 *μ*g/mL of SP-ZnONPs, it increases lactate dehydrogenase activity. A drastic dose-dependent increase in the LDH activity was evidenced in A549 cell lines after exposing to the SP-ZnONPs (Figure 14). Treated cells show higher significance compared with control cells (*P* < 0.0001).

## 4. Discussion

Lung cancer is one of the leading causes of death among all cancers. A variety of treatment strategies including surgery, chemotherapy, radiation therapy, and targeted therapy have been followed; however, the success rate is low. Green-synthesized nanoparticles are being actively explored as an anticancer drug. Especially, the potential of anticancer activity of ZnONPs has been thoroughly investigated.

ZnONPs nanoparticles have been established as an anticancer drug [19–21] because of their selective killing efficiency on proliferating cell lines [4, 22, 23]. *Solanum procumbens* has been extensively used in folk medicine in South East Asian countries. Therefore, we synthesized ZnONPs using *Solanum procumbens* extract. Further, we evaluated the synthesized SP-ZnONPs as an antilung cancer drug. The absorbance of the sample depends on several factors, such as band gap, oxygen deficiency, surface roughness, and impurity. The UV-Vis absorption spectrum of SP-ZnONPs shows an absorption maximum at 372 nm, which is blue shifted to 365 nm for bulk ZnONPs confirms the generation SP-ZnONPs [24].

The X-ray diffraction pattern of SP-ZnONPs is shown in Figure 2. The XRD peaks are located at angles (2*θ*) of 31.6881, 34.3314, 36.2027, 47.4636, 56.4647, 62.9138, 66.3306, 68.0310, 69.0153, and 76.8765, which correspond to the (100), (002), (101) (102), (110), (103), (200), (112), (201), (004), and (202) hkl planes of the SP-ZnONPs. The standard diffraction peaks show the hexagonal wurtzite structure of ZnONPs with space group p63mc. It is also confirmed by the JCPDS data (Card No: 36–1451) [25]. The average crystallite size of the sample was calculated using Debye–Scherrer's formula [26].

### 4.1. Average Crystallite Size *D* = k*λ*/*β*_Dcos*θ*

Where *D* is the size in nanometres, *λ* is the wavelength of the radiation (1.5406 Å for CuK*α*), *k* is a constant (0.94), and *β*D is the peak width at half-maximum in radian along (101) plane and in the Bragg's diffraction angle. The ZnONPs average particle size is 52 nm. To obtain the particle size information, the hydrodynamic diameter of green-synthesized SP-ZnONPs was determined using dynamic light scattering (Figure 3). The size of the SP-ZnONPs was measured at 154 nm; because the NPs were surrounded by water, the DLS particle size was larger than the XRD results. This is referred to as hydrodynamic size.

Figure 4 shows the photoluminescence spectra of green-synthesized SP-ZnONPs excited at 325 nm. The emissions were observed at 388, 421, 445, 459, 479, and 523 nm. The peak observed at 388 nm (near band edge), due to the free exciton-exciton collision process's radiative recombination [27]. The electron transition from the surface donor level of the zinc interstitials (Zni) to the top level of the valence band is responsible for the violet emission observed at 421 nm [28]. The three blue emission bands at 445, 459, and 479 nm correspond to the singly ionized Zn vacancies (VZn) [29]. The peak at 523 nm corresponds to the oxygen vacancies (Ov) [30].

SEM image of green-synthesized SP-ZnONPs is shown in Figure 5. From the image, it is clear that the SP-ZnONPs formed a spherical structure with agglomerated nanostructures due to the reduction of surface free energy by increasing their size and decreasing their surface area. The average particle size is found to be 30–60 nm, which is agreed well with the value determined by XRD. The IR spectrum of Solanum procumbens extract and SP-ZnONPs was shown in Figures 6(a) and 6(b), respectively. The broad peak at 3436 cm^−1^ in both Figures 6(a) and 6(b) confirms the presence of alcohol and phenolic OH groups; it is clearly understood that both phenols and alcohols present in the extract are caped with the nanoparticles. In addition, the peak at 495 cm^−1^ in the Figure 6(b) confirms the presence of SP-ZnONPs because the peak between 400 and 600 cm^−1^ regions responsible for stretching frequency of Zn–O bond in ZnONPs [31]. Most importantly, the peaks responsible for different functional groups such as -N-H and -C=*O* in the extract as shown in Figure 6(a) are completely disappeared in the case of SP-ZnONPs as shown in Figure 6(b). It clearly indicates that the compounds containing both alcoholic and phenolic OH groups in the extract are responsible for the generation of ZnONPs and remaining compounds present in the extract are leaching out while giving repeated washings.

Cytotoxic nature of the synthesized nanoparticles was evaluated by MTT assay (Figure 7). The cell viability was evaluated after treatment with SP-ZnONPs. In both the assays, the nanoparticle concentrations ranging between 5 and 200 *μ*g/mL were used against A549 cell lines. The results of cell viability assay correlated well with the cytotoxic assay (Figure 8). IC_50_ of the SP-ZnONPs was calculated to be 61.28 *μ*g/mL for MTT assay and 60 *μ*g/mL for cell viability assay.

The morphological changes during the cell death induced by SP-ZnONPs were evaluated by phase contrast microscopy. It was found that there is a dose-dependent reduction in the cell number; the optimized dose range is between 50 and 70 *μ*g/mL. When compared with control, drastic changes in the cellular morphology were also observed (Figures 9(a)–9(e). The cells were rounded up the sign of detachment from the substrate, which is an evidence for the morphologic hallmarks of apoptosis [32–34]. Integrins are involved in cell-matrix interaction through focal adhesion and linked kinases. Induction of apoptosis led to inactivation of focal adhesion [35] and linked kinases [36]. Overall, it could be concluded that the SP-ZnONPs cause cell deaths in the lung cancer cells through the apoptosis. Therefore, to confirm the apoptosis, induction AO/EB dual staining was carried out. Acridine orange stain has the propensity to penetrate into the normal and early apoptotic cells where the cell membrane is intact. It gives a fluorescent green colour upon binding to the DNA. On the other hand, ethidium bromide stain can only damage cells and gives orange red colour fluorescence when bound to the DNA [37]. The fluorescent images (Figure 10) indicate that the SP-ZnONPs induces a dose-dependent effect on lung cancer cells. At lower concentrations, viable and early apoptotic cells were observed with a scanty number of late apoptotic and necrotic cells, whereas at medium dose, the number of viable cells decreased with equal proportion of early and late apoptotic cells. Upon increasing the concentration, the number of apoptotic cells can be visualized with very rare viable cells. Overall, it is clear that SP-ZnONPs are effective in causing cell deaths by inducing apoptosis. Further, mechanism of induction of apoptosis was evaluated through the analysis of ROS because apoptosis is a main cause for the ROS increment. ZnONPs are well known for its efficacy in raising ROS [19]. Cellular ROS is capable of inducing cell cycle arrest, senescence, and subsequently apoptosis in cancer cells. Interestingly, ROS has been demonstrated to suppress metastasis also [38]. In the chemotherapy for cancer, exhausting antioxidant mechanism to elevate ROS through apoptosis is one of the effective strategies being followed [5]. SP-ZnONPs induced a significant increase in ROS through apoptosis in a dose-dependent manner. Even with 50 *μ*g/mL dose of SP-ZnONPs, there was a 1.5-fold increase in ROS, and with 70 *μ*g/mL dose, there was more than 3-fold increase in ROS level (Figure 11). It is clear that the apoptosis induced by SP-ZnONPs is an origin in the elevation of ROS level. NO is a negative regulator of apoptosis in a number of cell types including lung cancer. Hence, suppression of NO is very important for the activation of Bax through slug, especially in A549 cell lines [39]. In the current experiment, SP-ZnONPs significantly suppresses the NO level in A549 cell line in a dose-dependent manner (Figure 12). These results correlate well with the dose-dependent increase in apoptosis by SP-ZnONPs.

Lipid peroxidation is a result of oxidative stress, which leads to breakage of lipids. Ultimately, lipid peroxidation can lead to alterations in the fluidity and permeability of membranes since membranes are made of lipid bilayers and thus can cause loss of cellular integrity [40]. Furthermore, the end products of lipid peroxidation can also induce apoptosis [41]. Results indicate that SP-ZnONPs are effective in inducing lipid peroxidation in a dose-dependent manner (Figure 13). Therefore, it is reasonable to conclude that SP-ZnONPs-mediated lipid peroxidation caused apoptosis in lung cancer cells. The presence of lactate dehydrogenase enzyme (LDH) in assay medium indicates that the cells undergo lysis. Estimation of LDH for the doses 50, 60, and 70 *μ*g/mL of SP-ZnONPs revealed that the nanoparticles increase the LDH to a greater extent in a dose-dependent manner. Approximately 40-fold increase in LDH was seen with 70 *μ*g/mL of SP-ZnONPs treatment. This is a strong proof that the green-synthesized nanoparticles are able to induce cell death in A549 cancer cell lines.

In conclusion, SP-ZnONPs effectively induced apoptosis in A549 lung cancer cell line with the IC_50_ value of 61.28 *μ*g/mL. Further, SP-ZnONPs caused detachment and rounding up of cell lines. Apoptosis induction by the green-synthesized nanoparticles was confirmed by AO/EB dual staining. The apoptosis was mediated by elevated ROS generation, which further caused lipid peroxidation and resulted in induction of apoptosis. Therefore, SP-ZnONPs can be used for the treatment of lung cancer. However, further *in vivo* studies are required to validate the clinical application of the nanoparticles.

## Figures and Tables

**Figure 1:** UV-Visible absorbance spectrum of SP-ZnONPs.

**Figure 2:** X-ray diffraction patterns of SP-ZnONPs.

**Figure 3:** DLS spectrum of SP-ZnONPs.

**Figure 4:** PL spectrum of SP-ZnONPs.

**Figure 5:** SEM image of SP-ZnONPs.

**Figure 6:** (a) FTIR spectrum of Solanum procumbens extract. (b) FTIR spectrum of SP-ZnONPs.

**Figure 7:** Cytotoxicity of SP-ZnONPs on A549 cell line. The lung cancer cells were treated with 5, 10, 15, 20, 25, 30, 35, 40, 45, 50, 55, 60, 75, 100, 150, and 200 *μ*g/mL concentrations of nanoparticles. MTT assay was performed to determine the toxicity of nanoparticles.

**Figure 8:** Cell viability measured with trypan blue exclusion assay. 10–100 *μ*g/mL concentration of SP-ZnONPs was treated with A549 cell lines.

**Figure 9:** Phase contrast microscopic images of SP-ZnONPs-treated A549 cell lines. (a) Control, (b) 50 *μ*g/mL, (c) 60 *μ*g/mL, (d) 70 *μ*g/mL, and (e) standard drug (cisplatin).

**Figure 10:** Analysis of apoptosis by AO/EtBr staining method. (a) Image of untreated A549 cell line; (b) image of the 50 *μ*g/mL of SP-ZnONPs-treated A549 cell line; (c) image of the 60 *μ*g/mL of SP-ZnONPs-treated A549 cell line; (d) image of the 70 *μ*g/mL of SP-ZnONPs-treated A549 cell line. VC: viable cells; EA: early apoptotic cells; LA: late apoptotic cells; NC: necrotic cells.

**Figure 11:** Percentage of ROS release in A549 cell line after treated with SP-ZnONPs.

**Figure 12:** Concentration of NO in A549 cell line after treatment of various concentrations of SP-ZnONPs.

**Figure 13:** Concentration of lipid peroxidation level in A549 cell line after treatment of various concentrations of SP-ZnONPs.

**Figure 14:** LDH assay in A549 cell line after treatment of various concentrations of SP-ZnONPs.

## Data Availability

The research data used to support the findings of this study are included within the article.
